# Correlation between the Treg/Thl7 Index and the Efficacy of PD-1 Monoclonal Antibody in Patients with Advanced Non-Small-Cell Lung Cancer Complicated with Chronic Obstructive Pulmonary Disease

**DOI:** 10.1155/2022/2923998

**Published:** 2022-07-08

**Authors:** Xiaoyu Wang, Xinyuan She, Wei Gao, Xing Liu, Bin Shi

**Affiliations:** ^1^Department of Respiratory Medicine, The Affiliated Suqian Hospital of Xuzhou Medical University, Suqian, 223800 Jiangsu, China; ^2^Department of Pathology, The Affiliated Suqian Hospital of Xuzhou Medical University, Suqian, 223800 Jiangsu, China

## Abstract

**Objective:**

It was to explore the correlation between regulatory T cells (Treg)/T helper cell 17 (Thl7) and the efficacy of receiving a programmed death protein-1 (PD-1) monoclonal antibody (mAb) in patients with advanced non-small-cell lung cancer (NSCLC) complicated with chronic obstructive pulmonary disease (COPD).

**Methods:**

The research subjects were 82 patients who were clinically evaluated and treated in the Respiratory Department of Suqian Hospital connected with Xuzhou Medical University from January to December 2021. All of the patients were given PD-1 immunotherapy, and 50 healthy people were chosen as the control group. Classification was carried out according to tumor type and tumor stage. The levels of Th17 and Treg/Th17 in the peripheral blood of patients with different tumor-node-metastasis (TNM) stages and different types were compared, and the immune function, lung function (forced expiratory volume in one second/forced vital capacity (FEV1%/FVC), FEV1%, and FVC), and changes in inflammatory factors were compared before and after treatment. The levels of interleukin (IL)-17, IL-6, tumor necrosis factor (TNF)-*α*, and transforming growth factor (TGF)-*β* were compared between the two groups. The correlation between Th17 cells and Treg cells in the peripheral blood of patients with NSCLC complicated with COPD was analyzed.

**Results:**

After treatment, the levels of IL-17, IL-6, TNF-*α*, and TGF-*β* in patients with NSCLC combined with COPD were notably superior to those in the control group (*P* < 0.05). The immune function and lung function of the patients were improved after treatment. There were 43 cases of squamous cell carcinoma, 30 cases of adenocarcinoma, and 9 cases of large cell carcinoma. The proportion of Th17 cells to CD4+ T cells in the blood of the three types of patients and the proportion of CD4^+^CD25^Hi^CD127^Lo^ regulatory T cells to CD4+ lymphocyte cells in Treg cells showed no considerable difference among the different case types (*P* > 0.05). No considerable difference was indicated in Treg/Th17 in peripheral blood between stage IIIB and stage IV lung cancer patients (*P* > 0.05). A positive linear correlation was revealed between Th17 cells and Treg cells in the peripheral blood of patients with NSCLC combined with COPD, *R* = 0.26, *P* = 0.039.

**Conclusion:**

Treg and Th17 cells were shown to be much higher in lung cancer patients with COPD, which could lead to immunosuppression and tumor growth. PD-1 therapy for NSCLC has demonstrated efficacy and can improve patients' immunological state while being extremely safe.

## 1. Introduction

Lung cancer is a respiratory malignancy with high morbidity and mortality worldwide. Eighty-five percent of lung cancer patients have non-small-cell lung cancer (NSCLC), most of whom are diagnosed at an advanced stage. In 2016, 162,510 people died of lung cancer in the United States. Lung cancer has also become the cause of death of malignant tumors in China, and its morbidity and mortality are also increasing [1, 2]. At the individual level, there are several reasons for the disease, including smoking, environmental pollution, and occupational exposure. The patient can experience dyspnea, weight loss, hemoptysis, loss of appetite, and other symptoms. The patient will have severe mental pain, depression, anxiety, and fear, and the patient's quality of life will be greatly reduced. The main cause of lung cancer is smoking [3, 4]. Chronic obstructive pulmonary disease (COPD) is a common respiratory condition among the elderly that is linked to lung cancer incidence and patient symptom reports. COPD is becoming more common as economic development, and people's living standards increase at a rapid pace. According to the World Health Organization (WHO) survey, the mortality rate of COPD occupies fourth place in the time, and the prevalence in the elderly in China is roughly in the range of 6.5-8.5%, with a high patient rate of ten. Male COPD patients with moderate or heavy smoking and female COPD patients with smoking and occupation are also at high risk of lung cancer. Most elderly COPD patients with lung cancer have advanced cancer when diagnosed, and some patients cannot tolerate chemotherapy due to ventilatory dysfunction and pulmonary disease [5, 6]. COPD is an independent risk factor for lung cancer, and the incidence in lung cancer patients with COPD is five times higher than that in smokers with normal lung function [7–9]. Symptoms of many patients include dyspnea, cough, and sputum, which seriously affect patients' lives, and these symptoms also bring great trouble to patients' breathing [10–13].

Patients with NSCLC combined with COPD have ventilation disorders and poor lung functional reserve, and some patients are likely to lose the opportunity for surgery and chemotherapy due to delayed diagnosis, which requires many new forms of research and application in the treatment of NSCLC [14]. In addition to surgery, chemotherapy, radiotherapy, and targeted therapy, the treatment of NSCLC also includes immunotherapy. In recent years, immunotarget inhibitors have emerged as a new approach for NSCLC treatment [15, 16]. Conventional drugs for the treatment of lung cancer generally act directly on tumor cells to kill them. Immunosuppressants mainly block the inhibition and mutual ligand expressed on T cells to block the pathway at the immune checkpoint in the tumor microenvironment to stimulate the function of tumor-specific T cells [17, 18]. Endogenous antitumor immunity was enhanced, and antitumor ability was enhanced. PD-1 and programmed death-ligand 1 (PD-L1) inhibitors are used in the second-line treatment of NSCLC, and studies have shown that these inhibitors can be used as second-line treatments for advanced NSCLC [19, 20]. However, there are still some disadvantages; the side effects of drugs still exist, and the cure rate is only 18%, so it is particularly important to know which patients can benefit from immunotherapy [21]. Helper T cell 17 (Th17) is a subpopulation of CD4+ T lymphocytes other than Th1 and Th2 that are capable of independent regulation and differentiation mechanisms. Th17 cells are a new leukocyte differentiation antigen CD4 helper T cell subgroup that secretes IL-17 and plays a certain role in the process of tumor cases, infectious diseases, and autoimmune diseases [22]. Different from helper T cells, Treg cells play an inhibitory role in antitumor immunity, are responsible for the negative regulation of collective immune function, and can induce an immune response by inhibiting antitumor activity in the body. Under normal circumstances, Treg and Th17 cells maintain a balance. During differentiation, Treg and Th17 cells fight against each other. If cell differentiation of the inflammatory molecule Th17 is enhanced, Treg/Th17 imbalance will be caused, and the autoimmune system will be damaged, resulting in transplant rejection. Proinflammatory Th17 cells and anti-inflammatory Tregs work together to keep the body in balance, which is important for immune stability. An aberrant immune response results from the formation of an inflammatory response, and variations in Treg cell expression/Th17 cells alter the airway response. In recent years, it has become a hot topic to fully and deeply understand the differentiation and regulation mechanism of Treg and Th17 cells and to search for the role of these two cells in the development of related diseases. An imbalance between Treg and Th17 cells exists in autoimmune diseases and plays an important role in the immune response of cells. Treg and Th17 imbalance is closely related to the development and treatment of malignant tumors [23, 24]. In-depth study of Treg and Th17 indicators in advanced NSCLC patients could provide new methods for new anti-inflammatory analysis and immunotherapy, as well as new strategies for tumor treatment.

With the rapid development of biotechnology, the immune system has become increasingly recognized by people, and the use of immunotherapy for tumors has become a new form. In clinical application, the comprehensive tumor treatment system also occupies an important position, but the side effects after treatment have not been eliminated. It is also necessary to study Treg/Thl7 and (PD-1) monoclonal antibody (mAb) in the treatment of NSCLC complicated with COPD. Based on this, qualified patients with advanced NSCLC were included to explore the efficacy of the Treg/Thl7 index and (PD-1) mAb in the treatment of NSCLC, hoping to improve the recognition rate of patients with early lesions and provide a basis for screening and prediction of clinical immunotherapy.

The paper's organization paragraph is as follows: The materials and methods is presented in Section 2.  Section 3 analyzes the results and discussion of the proposed work.  Section 4 discusses the discussion of the paper. Finally, in Section 5, the research work is concluded.

## 2. Materials and Methods

### 2.1. The Research Objects

A total of 82 patients clinically diagnosed and treated in the Respiratory Department of Suqian Hospital affiliated with Xuzhou Medical University from 2021 January to December 2021 were selected as the research subjects. All patients received PD-1 immunotherapy for advanced NSCLC, and their clinical data were retrospectively analyzed. There were 17 females and 65 males, ranging in age from 45 to 72 years, with an average age of 54.62 ± 9.31 years. This experiment was approved by the ethics committee of Suqian Hospital affiliated with Xuzhou Medical University, and all patients and their families gave informed consent.

#### 2.1.1. Inclusion Criteria

- Long-term patients in our hospital
- Detailed information of inpatients (including age, sex, previous medication history, and disease history)
- Patients diagnosed with advanced NSCLC complicated with COPD by histological and imaging examinations, while disease progression cannot be tolerated after the failure of standard treatment, such as chemotherapy, targeted therapy, and immunotherapy other than targeting PD-1/PD-L1
- Patients with no other mental diseases
- Patients with good understanding and communication skills
- Advanced NSCLC patients without other treatment
- Patients with measurable lesions that met the *Response Evaluation Criteria in Solid Tumors 1.1* (RECIST 1.1)

#### 2.1.2. Exclusion Criteria

- Patients who did not agree to participate in this research
- Incomplete case data
- Patients with long-term use of hormones or hematopoietic factors
- Patients with acute or chronic inflammation (human immunodeficiency virus and hepatitis)
- Patients suffering from mental illness
- Patients with previous or existing autoimmune disorders
- Patients with pulmonary interstitial lesions

### 2.2. The Research Methods

All patients immunized with mAb to PD-1 underwent routine blood and biochemical tests one week before treatment and were divided into sintilimAb, toripalimAb, pembrolizumAb, and nivolumAb groups according to the type of PD-1 mAb.

SintilimAb treatment: a 3-week cycle of 200 mg drops of vein injection

ToripalimAb treatment: a 2-week cycle of 3 mg/kg drops of vein injection

PembrolizumAb: a 3-week cycle of 2 mg/kg drops of vein injection

NivolumAb: a 2-week cycle of 3 mg/kg drops of vein injection

Patients were divided into first-line, second-line, and ≥ third-line groups according to the number of lines received by PD-1 mAb. Patients were rolled into two groups regarding whether they smoked. Patients were rolled into two groups regarding whether there were immune-related adverse reactions.

According to tumor types, patients were classified into large cell carcinoma, adenocarcinoma, and squamous cell carcinoma groups. The tumor was stage IIIB or IV.

### 2.3. Experimental Reagents and Instruments

Flow cytometry was purchased from American BD, and the analysis software was *Diva*. 2IL-17A-APC antibody, antihuman Foxp3-PE antibody, film-breaking agent, and staining agent were purchased from the American eBioscience. APC-labeled mouse antihuman CD25, RPMI-1640 medium, hemolysin, and IL-17 mAb reagent were purchased from BD, USA. Ionomycin and phorbol 12-myristate 13-acetate (PMA) were purchased from the Sigma, USA. The 1% paraformaldehyde and lymphocyte isolate (Ficoll isolate) were purchased from Huajing Biotechnology. A medical centrifuge (KDC-1044) was purchased from USTC Innovation Co., Ltd. A waterproof constant temperature incubator (GSP-9050MBE) was purchased from Shanghai Boxun Industrial Co., Ltd. Medical Equipment Factory. A thermostatic oscillator was purchased from Shanghai Yuejin Medical Device Co., Ltd. A microplate reader was purchased from Tecan Austria.

### 2.4. Th17 and Treg Cells Detected by Flow Cytometry

Flow cytometry detection of Th17 cells referred to the detection of peripheral blood mononuclear cells, including monocytes and lymphocytes. Fifty healthy subjects and lung cancer patients were selected to take 5 mL venous blood and 2 mL separated serum at -20°C in the morning for use in an enzyme-linked immunosorbent assay (ELISA). Then, 3 mL was used for ethylenediaminetetraacetic acid (EDTA) anticoagulation. Two milliliters of peripheral anticoagulant blood was collected from lung cancer patients, diluted with phosphate-buffered saline (PBS) buffer of the same amount, and then mixed gently. The centrifuge tube was filled with ten milliliters of lymphocyte separation solution, and then PBS-diluted peripheral blood was deposited onto the liquid surface of the lymphocyte separation solution. It was ensured that there was a clear interface between the liquid level, and after centrifugation for 20 min at 2,000 r/min and stratification, the lower layer was displayed for red blood cells and neutrophils, the upper layer was displayed for plasma and platelets, and the intermediate layer was a cloud of mononuclear cells. The cloud layer was slowly inhaled in another 15-mL centrifuge tube, and then five times the PBS buffer was added. After mixing, centrifugation was conducted for 10 min at 1,000 r/min, and the obtained precipitate was mononuclear cells, which were counted under the microscope, and the cell density was adjusted to 2 × 10^6^ per mL.

One millimeter of lymphoid tissue was added to 1 mL Roswell Park Memorial Institute (RPMI1640) medium and filtered through a 200-mesh steel mesh. The cell density was adjusted to 1 × 106/mL, and then the final concentration of phorbol ester was added to 100 ng/mL, the final concentration of ionomycin was added to 1 mg/L, and the final concentration of monomycin was added to 2 mL/L. The cells were placed in an incubator with 5% CO_2_ at 37°C and stimulated for 6 hours.

Intracellular antibody labeling was performed as follows. The stimulated cells were fixed with 1% paraformaldehyde for 15 minutes, washed with PBS, and centrifuged for 5 min at 1,500 r/min, and the supernatant was removed. Then, phycoerythrin (PE)-labeled mouse antihuman CD8 antibody and rat antihuman CD3 antibody labeled with fluorescein isothiocyanate (FITC) were added, incubated at room temperature for 20 min in the dark, washed again with PBS, and centrifuged for 5 min at 1,500 r/min, and then the supernatant was discarded. Then, 200 *μ*L of film breaker was added, incubated at room temperature for 20 min in the dark, centrifuged, added to APC-labeled mouse antihuman IL-17 antibody, incubated for 20 min, washed with PBS, and centrifuged for 5 min at 1,500 r/min. Then, the supernatant was superfluous. Then, 300 *μ*L PBS was added to suspend the cells. The cells were transferred to a special flow cytometer tube, away from light standby, for analysis.

### 2.5. Flow Cytometry Detection of the Proportion of CD4^+^CD25^Hi^CD127^Lo^ Regulatory T Cells in CD4+ Lymphocytes

One hundred microliters of anticoagulant whole blood from patients in observation group and healthy controls was added to the flow tube. Antibodies against CD4-FITC, CD25-APC, and CD25-APC were added to each detection tube according to the operation steps and then mixed and incubated at room temperature for 20 min. Two milliliters of hemolysin was added, fully mixed, and then incubated at room temperature for 10 minutes. After the red blood cells were fully lysed, PBS was added to each tube twice for washing. The lysed red blood cells were obtained by centrifugation for 5 min at 1,500 r/min. In the detection before the machine, 200 *μ*L PBS was added to each tube for blending. Then, *CellQuest* was used to analyze the results, and the percentage of CD4^+^CD25^Hi^CD127^Lo^ regulatory T cells in CD4+ lymphocyte cells in Treg cells was expressed.

### 2.6. Serum IL-17 Concentration Detected by ELISA

The concentration of IL-17 in serum was detected by a double-antibody sandwich. First, all reagents were restored to room temperature. Fifty milliliters of concentrated IL-17 solution was prepared, and 950 mL of double distilled water was added to it and fully mixed for later use. Then, 5 mL of IL-7 analysis buffer stock was added to 95 mL of double steam water and mixed well. For antibody preparation, 60 *μ*L of IL-17 enzyme antibody was added to 5.94 mL of dilution analysis buffer for later use. Then, 11.94 mL of the prepared solution was added to 60 *μ*L of streptavidin-HRP, which was prepared half an hour before the addition. The standard il-17 solution was then prepared, and 400 *μ*L of double distilled water was added to the il-17 powder to resuscitate to prepare a standard il-17 concentrate of 200 pg/mL. Seven tubes were labeled as 1-7, and 225 *μ*L dilution analysis buffer was added to them. A standard concentrate of 200 pg/mL RGF-*β*1 (225 *μ*L) was added to tube no. 1 and mixed. Standard curves with concentrations of 100, 50, 25, 12.5, 6.3, 3.1, and 1.6 pg/mL were successively prepared, and diluted analytical buffer was selected as a blank.

The specific operation steps are as follows. First, the 96-well plate was washed twice with buffer solution on the automatic plate washing machine and then dried. Seven standard series solutions were added to the wells, and 50 *μ*L of analysis buffer was added to the other wells. Then, 50 *μ*L of enzyme antibody was added to each well, shaken, incubated for 2 h at 100 r/min, and then washed 4 times. After drying, 100 *μ*L of streptavidin-HRP was added, incubated for 1 h by shaking for 100 r/min, washed, and dried again. Then, 100 *μ*L chromogenic agent was added to each well and incubated for 10 min at room temperature. Finally, 100 *μ*L stop solution was added. After mixing, the optical density was determined at 450 nm using a microplate reader to calculate the concentration of IL-1. IL-6 was determined using the same method.

### 2.7. Serum TGF-*β* Concentration Detected by ELISA

TGF-*β*concentrations in serum were also measured using a double-antibody sandwich ELISA. All reagents were first brought to room temperature. Fifty milliliters of TGF-*β*concentrate were made, and 950 milliliters of double-steamed water were added and thoroughly mixed before being used. Then, 5 mL of TGF-*β* analysis buffer stock was added to 95 mL of double-steamed water and mixed well. For antibody preparation, 120 *μ*L TGF-*β* enzyme antibody was added to 11.88 mL dilution breakdown buffer for later use. Then, 11.88 mL streptavidin-HRP was added to 120 *μ*L streptavidin-HRP, and the solution was organized half an hour before the addition. Then, a TGF-*β* standard solution was prepared, 400 *μ*L double steam water was added to the TGF-*β* powder, and 4,000 pg/mL TGF-*β* standard ponder was prepared after resurgence. Seven tubes were labeled as 1-7, and 225 *μ*L dilution analysis buffer was added to them. A standard solution of 2,000 pg/mL was prepared by adding 225 *μ*L of 4,000 pg/mL RGF-*β*1 standard concentrate into a no. 1 tube. Then, it was added to a no. 2 tube, mixed evenly, and successively used to prepare standard curves with concentrations of 2,000, 1,000, 500, 250, 125, 63, and 31 pg/mL. Dilution analysis buffer was selected as a blank.

First, the sample was pretreated. The sample was diluted at a ratio of 1 : 10. 180 *μ*L dilution analysis buffer was added to 20 *μ*L sample, and 20 *μ*L1N hydrochloric acid solution was added, mixed. After incubation for 1 h, the sample was neutralized with 20 *μ*L of 1 N NaOH in a 96-well plate. The plate was washed twice with buffer solution on an automatic plate washing machine and then patted dry. The wells were filled with seven standard series solutions, and the rest went into the analysis buffer. Then, 60 *μ*L analytical buffer solution was added to each well, and 40 *μ*L pretreated samples were added in turn, shaken, and incubated at 100 r/min for 2 h. The automatic plate washing machine was employed to wash it 5 times, patted dry, added to 100 *μ*L of enzyme antibody, shaken again for 100 r/min, incubated for 1 h, washed 5 times, and patted dry again. Streptavidin-HRP (100 *μ*L) was added to each well, shaken, incubated at 100 r/min for 1 h, washed 5 times, and patted dry again. Then, 100 *μ*L chromogenic agent was added to each well and incubated at room temperature for 30 minutes. Then, 100 *μ*L stop solution was added and mixed well. A microplate reader was employed to determine the optical density at 450 nm, and the concentration of TGF-*β* was calculated. The same method was used to determine TGF-*α*.

### 2.8. Statistical Methods

Excel 2007 and SPSS 25.0 (SPSS Inc., Chicago, IL, USA) were used to input the collected data for statistical analysis. Analysis of variance was adopted to compare the correlation between Th17 cells and Treg cells*. CellQuest* was employed to analyze the results, and Th17 cells were expressed as a percentage. The mean ± standard deviation( $\bar{x}$ ± *s*) was used to represent the measurement data conforming to a normal distribution. ANOVA was used to represent Th17 cells and Treg cells among lung cancer groups with different stages and types, and frequency and frequency (%) were used to represent the nonconforming count data. The correlation between Th17 cells and Treg cells was analyzed by Pearson correlation analysis. The counting data were tested by *χ*^2^. The difference was substantial at *P* < 0.05.

## 3. Results and Discussion

### 3.1. General Information

Among the 82 patients selected, 65 were male, accounting for 79.27%, and 17 were female, accounting for 20.73% (Table 1). There were 31 patients in stage IIIB, accounting for 37.80%, and 51 patients in stage IV, accounting for 62.20%. There were three tumor types, including 43 cases of squamous carcinoma (52.44%), 30 cases of adenocarcinoma (36.59%), and 9 cases of large cell carcinoma (10.98%). The 52 cases of smoking patients accounted for 63.41% higher than that of nonsmoking patients. There were 25 cases with immunotoxic reactions (30.49%) and 57 cases without immunotoxic reactions (69.51%).

### 3.2. Ratio of Th17 Cells in Peripheral Blood

Eighty-two patients with NSCLC combined with COPD were the observation group, and normal healthy people were the control group.  Figure 1 shows that the proportion of Th17 cells in the peripheral blood of patients in observation group was notably superior to that in the controls (*P* < 0.01). Treg/Th17 in the peripheral blood of patients decreased remarkably versus controls (*P* < 0.05).

### 3.3. Comparison of Th17 and Treg/Th17 Cells of Patients with Different Case Types

Among the 82 subjects, there were 43 cases of squamous cell carcinoma, 30 cases of adenocarcinoma, and 9 cases of large cell carcinoma (Figure 2). There was no considerable difference among different case types in the proportion of Th17 cells in CD4+ T cells in the blood of the three types of patients and the proportion of CD4^+^CD25^Hi^CD127^Lo^ regulatory T cells in CD4+ lymphocyte cells of Treg cells (*P* > 0.05).

### 3.4. Comparison of Peripheral Blood Th17 and Treg/Th17 in Patients with Different TNM Stages

There was no considerable difference in the proportion of Th17 cells to CD4+ T cells in the peripheral blood of patients with stage IIIB and stage IV lung cancer (Figure 3), and there was no great difference in the proportion of CD4^+^CD25^Hi^CD127^Lo^ regulatory T cells to CD4+ lymphocyte cells in Treg cells (*P* > 0.05). There was no considerable difference in Treg/Th17 in peripheral blood between stage IIIB and stage IV lung cancer patients (*P* > 0.05).

### 3.5. Correlation Analysis of Th17 Cells and Treg Cells of Lung Cancer Patients with COPD

The correlation between Th17 cells and Treg cells in the peripheral blood of patients with NSCLC complicated with COPD was analyzed. The results are shown in Figure 4, showing a positive linear correlation between the two, *R* = 0.26 and *P* = 0.039.

### 3.6. Comparison of Immune Function before and after Treatment

In Figure 5, CD4+ and CD4+/CD8+ were notably superior to before treatment, while CD8+ was greatly inferior to before treatment. The cellular immune indexes of patients before and after treatment were compared, and the difference was substantial (*P* < 0.05).

### 3.7. Pulmonary Function Changes before and after Radiotherapy

The FEV1%/FVC, FEV1%, and FVC of patients before and after chemotherapy were compared and analyzed (Figure 6), and the difference was substantial one month after radiotherapy compared with that before radiotherapy (*P* < 0.05). There was no considerable difference in FEV1%/FVC of patients two weeks after radiotherapy compared with that before radiotherapy (*P* > 0.05), but there were considerable differences in FEV1% and FEV (*P* < 0.05). After receiving radiotherapy, the lung function of patients showed varying degrees of change, with some changes in lung function, and some indexes had considerable differences relative to those before radiotherapy (*P* < 0.05).

### 3.8. Comparison of MVV/MEF before and after Radiotherapy

In Figure 7, MVV and MEF were changed after two weeks and one month of treatment compared with those before treatment, and pulmonary function improved remarkably (*P* < 0.05).

### 3.9. Comparison of the Peripheral Blood Cytokines IL-17, IL-6, TNF-*α*, and TGF-*β*

The levels of IL-17, IL-6, TNF-*α*, and TGF-*β* in the peripheral blood of lung cancer patients in observation group and control group were compared (Figure 8), and those in lung cancer patients with COPD were notably superior to those in control group (*P* < 0.05).

## 4. Discussion

COPD is a widespread respiratory disease with a high mortality rate, affecting more than 5% of the world's population. Cough and sputum are the most common clinical symptoms of COPD and lung cancer, and misdiagnosis and missed diagnoses are common during the diagnosis and treatment process [25]. Immunosuppressants have been applied to treat NSCLC and have brought some benefits to patients. Clinically, the lung function and immune function of patients with NSCLC complicated with COPD will decline to varying degrees, as will their immunity [26, 27]. Clinical data showed that patients with NSCLC complicated with COPD had different degrees of decline in lung function after receiving radiotherapy, and patients received different doses of radiotherapy. In this study, patients with advanced NSCLC complicated with COPD were treated with PD-1 and Treg/Th17 cells. Comparative investigation of the results of patients before and after radiotherapy showed that the lung function of various patients showed different degrees of change after radiotherapy. The change in lung function was more dramatic than the change before treatment, and some lung function indicators were significantly different from those before radiotherapy, with statistical significance (*P* < 0.05). In many studies of COPD, FEV1%/FEV and FEV1% are the primary evaluation indexes. Studies have shown that the diagnostic rate of the lung function index of FEV1%/FVC, FEV1%, and FVC is more than 95%. There was a large difference in the therapeutic effect of NSCLC between smokers and nonsmokers. Smokers had a higher mutation load, and the response to immune target inhibitors was also enhanced. PD-1 has a poor therapeutic effect on smokers, which also shows that smoking history can be an effective predictor [28, 29].

Immunotherapy for NSCLC has taken a new turn with the introduction of immunosuppressive medicines. These medications have few side effects, are well tolerated, and are frequently utilized in the treatment of tumors. In this study, a PD-1 mAb was used to treat NSCLC patients. CD4+ and CD4+/CD8+ were remarkably higher after treatment than before, while CD8+ was greatly inferior to before. The cellular immune indexes of patients before and after treatment were compared with those before treatment, and the difference was substantial (*P* < 0.05), indicating that PD-1 can improve the immune function of patients with NSCLC and has high clinical application value. This is consistent with many studies. PD-1 expression is one of the most widely used clinical markers for immunotherapy prediction, and the expression of PD-1 in solid tumor tissues monitored by histochemistry is associated with poor prognosis of gastric cancer, liver cancer, and cell carcinoma. Data suggest that patients with advanced NSCLC with high PD-1 expression respond better to pembrolizumAb treatment [30]. PD-1 mAb is effective in tumor immune escape due to its role in promoting tumor T cell apoptosis in both an independent and dependent manner. By altering the surrounding environment, cancer cells promote immune evasion, multiplication, and survival. PD-1 therapy's main goal is to stimulate T lymphocytes in the tumor microenvironment in order to establish tumor resistance [31, 32]. Gauvain et al. [33] looked at patients with NSCLC brain metastases who were given nivolumAb and found that the intracerebral control rate was 51%, indicating some safety. The level of Th17 cells increases to varying degrees in a variety of solid tumor tissues. In cancer diseases, the higher the TNM stage, the more obvious the increase in the level of Th17 cells. Th17 cells can secrete IFN-*ɤ* to a certain extent, which can play an antitumor role. Studies have shown that TGF-*β* can inhibit Th17 production and induce Treg cell formation in ovarian cancer cells. Th17 cells in tumor patients were greatly inferior to those in normal subjects, indicating immunosuppression in the tumor microenvironment. When the Treg level increases, antitumor immunity is suppressed, resulting in an imbalance in the Th17/Treg status in tumor patients [34]. Li et al. [35] discussed the relationship between TregFoxP3(+) and Th17 cells and the occurrence of lung cancer and showed that the ratio of TregFoxP3(+), Th17 and TregFoxP3(+)/Th17 in the peripheral blood of NSCLC patients was higher than that of healthy controls (*P* <0.05). The proportion of Th17 cells in NSCLC patients was positively correlated with the proportion of TregFoxP3(+) (*r* = 0.81, *P* < 0.05). In this study, the same results were obtained, and there was a positive linear correlation between Th17 cells and Treg cells in the peripheral blood of patients with NSCLC combined with COPD by Treg/Th17 ratio analysis after treatment in NSCLC patients, *R* = 0.26, *P* = 0.039. TGF-*β*, IL-17, and IL-6 levels were higher in NSCLC patients than controls. Patients with stage IIIB and IV disease showed significant improvement in lung function after PD-1 immunotherapy. It was concluded that the Treg/Th17 ratio was related to the stage of NSCLC, but there was no considerable difference between TNN stages in this study, and both stage IIIB and stage IV were probably advanced, so the difference was not significant. The patients' immunological indices improved after treatment. This also suggests that PD-1 immunotherapy influences the immune status of patients with advanced NSCLC.

## 5. Conclusions

The efficacy of Treg/Th17 and PD-1 monoclonal antibodies in the treatment of NSCLC in patients with NSCLC complicated with COPD was investigated. Treg and Th17 cells were remarkably higher, which may lead to immunosuppression and promote tumor formation in COPD patients with NSCLC. PD-1 treatment of NSCLC has clear efficacy and can improve the immune status of patients with high safety. The cytokine modulation of Treg and Th17 cells may be linked to the Treg/Th17 ratio imbalance in lung cancer patients. Furthermore, follow-up research can conduct in-depth studies on the imbalance of the Treg/Th17 ratio in the hopes of clarifying the relationship between many components in this process and providing more accurate data support for tumor cure.

## Figures and Tables

**Figure 1:** Comparison results of peripheral blood cells between the two groups. (∗ indicates considerable difference, *P* < 0.05).

**Figure 2:** Comparison of Th17 and Treg/Th17 cell proportions of patients with different case types.

**Figure 3:** Comparison of Th17 and Treg/Th17 cell proportions of patients with different TNM types.

**Figure 4:** Correlation between peripheral blood Th17 cells and Treg cells.

**Figure 5:** Comparison of immune function before and after treatment. (∗ indicates a substantial difference vs. before treatment, *P* < 0.05).

**Figure 6:** Comparison of FEV1%/FVC, FEV1%, and FVC before and after chemotherapy. (∗ indicates a substantial difference vs. before radiotherapy, *P* < 0.05).

**Figure 7:** Comparison of MVV and MEF before and after chemotherapy. (∗ indicates a substantial difference vs. before radiotherapy, *P* < 0.05).

**Figure 8:** Comparison of the cytokines IL-17, IL-6, TGF-*β*, and TGF-*α* in peripheral blood. (∗ indicates a substantial difference vs. before treatment, *P* < 0.05).

**Table 1:** General clinical characteristics of the patients.

	Total	Proportion	*P*
Gender	82	100%	0.812
Female	17	20.730	
Male	65	79.270	
Tumor staging			0.531
IIIB	31	37.800	
IV	51	62.200	
Tumor types			0.624
Adenocarcinoma	30	36.590	
Squamous cell carcinomas	43	52.440	
Large cell carcinoma	9	10.980	
Smoking			0.063
No	30	36.590	
Yes	52	63.410	
Immune toxicity and side effects			0.008
No	57	69.510	
Yes	25	30.490	

## Data Availability

The data used to support the findings of this study are available from the corresponding author upon request.
